RETRACTED

# Determinants of the Intention to Use Smart Healthcare Devices: A Framework and Public Policy Implications

**DOI:** 10.1155/2021/4345604

**Published:** 2021-11-05

**Authors:** Xifeng Lu, Junyi Hao, Biaoan Shan, Anwei Gu

**Affiliations:** ^1^School of Accounting, Jilin University of Finance and Economics, Changchun, China; ^2^School of Management, Jilin University, Changchun, China

## Abstract

Healthcare industry is strongly influenced by new digital technologies. In this context, this study creates a framework and explores determinants of the intention to use smart healthcare devices. Several factors were identified, including usefulness, convenience, novelty, price, technological complexity, and perceived privacy risks of smart devices. Based on the samples from China, we find that usefulness, convenience, and novelty have positive influences on the intention to use smart healthcare devices. However, technological complexity is negatively related to the intention to use smart devices. The results further extend previous researches in the area of the healthcare industry.

## 1. Introduction

In the past few years, digital technologies have developed quickly and are widely applied in many industries. These new emerging technologies, including cloud computing, big data analytics, Internet of Things, artificial intelligence, mobile communications, virtual reality, and machine learning, significantly influence our daily life and the global economy [1, 2]. Many novel products or services have been created and have strongly enhanced our life. There is no doubt that we have entered the era of digital economy. More and more industries will be impacted and changed by the promotion of emerging digital technologies [3, 4].

In the healthcare industry, the application of emerging digital technologies has dramatically changed the service modes; for example, telemedicine has improved the convenience of healthcare services [5]. Under the support of the Internet of Things, big data and mobile communications, smart medical service and management systems are developing fast. Various forms of smart healthcare devices for monitoring health and well-being across all ages begin to prevail in the healthcare industry [6]. The smart devices based on digital technologies can collect and analyze users' data and have effectively improved users' health management [7]. Therefore, this area is focused by a large number of entrepreneurs, investors, and healthcare professionals.

Because of its important value in the application of healthcare, smart devices based on new technologies have been concerned by existing researchers [8–10]. Literatures on this area mainly focus on three aspects. First, one major stream of existing studies explores the impact of various digital technologies on smart devices, for example, exploring the roles of Internet of Things and blockchain technology in the design of smart devices [7, 8]. Second, it examines the effect of smart healthcare devices on individuals' care and smart cities [11, 12]. Third, a few studies investigate the challenges faced by smart healthcare [13]. These researches have enriched the understanding of smart healthcare devices. However, smart devices are relatively novel to users and customers. It is an important topic to reveal the factors to improve the intention to use smart devices. Only few studies focus on this issue. We still know little about the determinants of the intention to use them.

RETRACTED

Based on the above, this study attempts to address this gap. A framework is established in this paper to reveal the determinants of the intention to use smart healthcare devices. We conduct surveys in many cities in China and investigate the factors influencing the acceptance of smart devices. By doing so, we contribute to the research area of smart healthcare and further improve the understanding of users' intention to accept smart healthcare devices. Also, the findings are beneficial for government to provide relative policies to support the development of smart healthcare devices industry.

This study is structured as follows: theory background and hypotheses are provided in Section 2; Section 3 introduces the methods used in this article; the results are shown in Section 4; theoretical and management implications are shown in Section 5; in Section 6, we draw conclusions of this article.

## 2. Theory Background and Hypotheses

### 2.1. Smart Devices

Internet of Things, machine learning, blockchain, and other emerging digital technologies create a lot of new business opportunities for individuals and organizations [1, 4, 14, 15]. In this context, various smart devices used to collect data and monitor users' health conditions are emerging in the healthcare industry [8–10]. Different from the ways of traditional healthcare, services based on these new devices are more convenient, smart, and functional.

Considering the innovativeness of these smart devices, researches in this area are still in the early stage. In conclusion, literatures on this topic mainly focus on the following aspects. First, one important stream studies the impact of various digital technologies on smart devices. They explore the roles of Internet of Things and blockchain technology in the design of smart devices [3, 8]. Second, many scholars explore the effect of smart healthcare devices on individuals' care and smart cities [11, 12]. Finally, a few studies investigate the challenges faced by smart healthcare and discuss future directions [13].

RETRACTED

Besides these, some researchers have analyzed the acceptance of smart devices. Because of the novelty of digital technologies, it is a crucial issue to improve the level of users' acceptance of smart devices. How to facilitate technology acceptance is not a new topic. Previous studies have concerned about it widely, such as the areas of information systems, technology management, and marketing management [12, 14]. The most discussed is the attribute of technologies, including technological complexity, novelty, and relationality [15]. However, only few studies have discussed the acceptance of smart devices. For example, Magni et al. [14] identified four antecedents of the intention to use wearable smarts, including organizational trust, hedonic motivations, privacy, and perceived usefulness. Yang et al. [16] revealed three important factors affecting the utilization of smart home services, including mobility, privacy risk, and trust in the product or service provider. Kim and Shin [17] identified several psychological determinants, such as affective quality, relative advantage, mobility, and availability. Little literature discusses the characteristics of customers. Park [18] discussed five factors, including satisfaction, flow state, enjoyment, usefulness, and cost. Obviously, existing studies do not consider the impacts of attributes of technologies and products, and individual characteristics on the acceptance in one framework.

In order to understand the acceptance of smart healthcare devices and reveal how to improve the intention to use the smart devices, we try to integrate the individual characteristics, technological characteristics, and the attributes of the products or services provided by smart devices. Specifically, we consider the usefulness, convenience, novelty, price of smart devices (attributes of products or services), technological complexity (technological characteristic), and perceived privacy risk (individual characteristic) in this study (see Figure 1). We will discuss them in the following parts.

### 2.2. The Attributes and Intention to Use Smart Healthcare Devices

According to the view of Magni et al. [14], usefulness is one of the antecedents for individuals to accept new technologies. Usefulness refers to users' perceived benefits of adopting technologies or devices. Formal scholars revealed that the usefulness and perceived benefits have a positive influence on adoption intentions [19]. For example, Kim, Mirusmonov and Lee [20] found that usefulness positively impacts on the intention to use mobile payment. Kuo and Yen [21] pointed out that usefulness has a positive effect on the intention to use 3G mobile services. Smart healthcare devices show important benefits on physical condition monitoring and health management [3]. Based on the above, we propose that usefulness is positively related to the intention to use smart healthcare devices.

RETRACTED

Hypothesis 1: usefulness is positively related to the intention to use smart healthcare devices.

Like usefulness, convenience is also an important attribute impacting the acceptance of new devices. Convenience is a combination of time and place utilities [20]. Only when technology or smart devices are easy to operate and make people's life convenient can users accept them. According to Berry et al. [22], time and effort will be saved if smart devices are convenient. Perceived convenience could be seen as an advantage. For smart healthcare devices with convenience, they are easier to operate. Just like Hsu and Chang [23] pointed out that convenience positively affects users' acceptance and use of IT, so this study proposes that convenience exerts a positive impact on the intention to use smart devices.

Hypothesis 2: convenience is positively related to the intention to use smart healthcare devices.

Novelty is one salient attribute of smart devices. It refers to the degree of newness in the market. High novel smart devices show significant innovativeness and big difference in the market [24]. This type of smart device is always related to radical innovation [25]. From the firm perspective, radical innovations will positively influence the outcome of organizations because it is beneficial to satisfy customer needs [26]. From the individual perspective, novel smart healthcare devices with new services contribute to attracting customers. Novel functions and services will facilitate grasping customer needs. Therefore, novelty strongly improves the intention to use smart healthcare devices.

Hypothesis 3: novelty is positively related to the intention to use smart healthcare devices.

Price is a sensitive factor, which determines the intention to use smart devices. Smart band is one type of typical healthcare device. It could monitor users' information such as electrocardiograms. This device is very popular among young users because of the low price. However, the price of some professional smart devices is often high, which are generally purchased and utilized by special medical institutions. Obviously, high prices create a threshold for users and will negatively impact the acceptance of these devices. Therefore, this study proposes the following hypothesis.

Hypothesis 4: price is negatively related to the intention to use smart healthcare devices.

RETRACTED

### 2.3. Technological Complexity and the Intention to Use Smart Healthcare Devices

Technological complexity refers to complex knowledge and skills for users. Sharma and Yetton [27] revealed that users are always more likely to reject to utilize the products or services with complex technology because technological complexity creates more obstacles to use. In this context, users always need assistant or technical support to operate complex technologies. Complexity is considered as a type of physical characteristic [28]. The high complex technology results in new products or services which are difficult to train, although it may improve new functions and more advanced skills are required for users. Antoniadis, Edum-Fotwe, and Thorpe [29] pointed out that complexity may increase the error rate of the system, such as causing delay. Therefore, technological complexity is strongly related to uncertainty to users [30]. Customers must frequently face and cope with the problem that may occur. Based on the above, we propose the following.

Hypothesis 5: technological complexity is negatively related to the intention to use smart healthcare devices.

### 2.4. Perceived Privacy Risk and the Intention to Use Smart Healthcare Devices

Existing researches have revealed that privacy risk is an important issue under the development of new digital technologies [31, 32]. In the research of Hiranandani [33], privacy is considered as a crucial dimension that cannot be ignored in the digital age. How to protect privacy has become a topic that must be coped with in the process of new technology development.

The services of smart healthcare devices are based on users' information. Therefore, perceived privacy risk always negatively influences the intention to use these smart devices. Magni et al. [14] find that privacy is a significant risk in the adoption of smart devices. Their study indicated that privacy is negatively related to the intention to use wearable devices. Obviously, perceived privacy risk of users negatively impacts the acceptance of smart healthcare devices. Therefore, we propose the following hypothesis.

Hypothesis 6: perceived privacy risk is negatively related to the intention to use smart healthcare devices.

## 3. Methods

### 3.1. Data Collection and Sample Characteristics

In order to text the hypotheses, a survey was considered and conducted during August and September, 2021. This survey was executed online. The formal survey was conducted in China. We collected samples from several cities, including Shanghai, Tianjin, Changchun, Zhengzhou, Wenzhou, and Shangqiu. These cities come from different areas of China, such as northeast area, central area, and eastern coastal area. In addition, the economy of some cities has developed well (e.g., Shanghai and Tianjin), while others have developed slowly (e.g., Changchun and Shangqiu). Therefore, the data collected from these cities indicate high representativeness.

RETRACTED

Finally, a total of 202 questionnaires were collected online. The characteristics of this sample are as follows (see Table 1).

### 3.2. Measurement and Reliability Analysis

This study utilizes Likert 5-point scale to measure the core variables. The items of core variables are shown as follows.

#### 3.2.1. Dependent Variable

The dependent variable is the intention to use smart healthcare devices. Based on the view of Magni et al. [14], three items are used to measure this variable (IU1-IU3). Two examples are “I really want to use these smart devices” and “I will buy these smart devices in the future.” The factor loading of items for the variable is more than 0.7. The Cronbach's alpha coefficient is 0.911.

#### 3.2.2. Independent Variables

The independent variables of this study contain attributes of the products or services provided by smart devices and individuals' characteristics.

The attributes include usefulness, convenience, novelty, price, and technological complexity. Drawing on the research of Alsabawy et al. [34], we ask subjects the usefulness provided by smart devices such as smart manometer and sphygmomanometer. Based on this study, the usefulness is measured by four items (US1-US4). Two examples are “using these smart devices allows me to know my physical condition more quickly” and “using these smart devices is beneficial for me to keep body healthy.” All the factor loadings of items for the variable are more than 0.7. The Cronbach's alpha coefficient is 0.925.

One item is used to measure the variable of convenience (CS: using these smart devices makes me feel very convenient).

According to Nieto and Santamaría [35], three items are developed to measure the novelty of products or services (NS1-NS3). Two examples are “these smart devices are special in the market” and “the services provided by these smart devices are relatively novel.” All the factor loadings of items for the variable are more than 0.7. The Cronbach's alpha coefficient is 0.905.

We also use three items to measure the price (ES1-ES3). Two examples are “the price of these intelligent medical devices is always unacceptable” and “these smart devices are less economical.” All the factor loadings of items for the variable are more than 0.7. The Cronbach's alpha coefficient is 0.952.

Based on the study of Sharma and Yetton [27], we utilize three items to measure technological complexity (TC1-TC3). Two examples are “these smart devices are difficult to operate” and “these smart devices involve many different technologies.” All the factor loadings of items for the variable are more than 0.7. The Cronbach's alpha coefficient is 0.917.

RETRACTED

Perceived privacy risk is used to reflect individual characteristics. According to Magni et al. [14], this study utilizes four items (PR1-PR4). Two examples are “using these smart devices makes me feel controlled” and “using these smart devices makes personal information risky.” All the factor loadings of items for the variable are more than 0.7. The Cronbach's alpha coefficient is 0.878.

#### 3.2.3. Control Variables

We set several control variables. First, we controlled the age of subjects (1, 30 years or below; 2, 30–40 years; 3, 40–50 years; 4, 50–60 years; 5, above 60 years). Second, work experience was controlled based on the years individuals have worked (1, 3 years or below; 2, 3–5 years; 3, 5–10 years; 4, above 10 years). Third, the family annual income was also set as a control variable (1, 30 000 RMB or below; 2, 30 000–60 000 RMB; 3, 60 000–100 000 RMB; 4, 100 000–150 000 RMB; 5, above 150 000 RMB). Fourth, we controlled individuals' educational background (1, high school or below; 2, junior college; 3, bachelor's degree; 4, master or Ph.D. degree).

## 4. Results

We first analyze the descriptive statistics. From Table 2, we can see the results. The mean and standard deviation are reasonable. The coefficients of Pearson correlation among core variables are also shown in the table. The results show that there are significant correlations among core variables. And then, multiple linear regression analysis (MLR) is utilized to examine the hypotheses of this study.

In order to test all the hypotheses, we established two models (see Table 3). Model 1 verified the influences of control variables on the intention to use smart healthcare devices while model 2 tests the effects of independent variables on the intention to use smart healthcare devices. The results show that the impacts of control variables on the intention to use smart devices are not significant.

From the results of model 2, the coefficient of usefulness is 0.371 (*p* < 0.0001). Therefore, Hypothesis 1, usefulness is positively related to the intention to use smart healthcare devices, is tested by samples. The coefficient of convenience is 0.319 (*p* < 0.0001). Hypothesis 2, convenience is positively related to the intention to use smart healthcare devices, is also supported by data. The coefficient of novelty is 0.143 (*p* < 0.0001). This result shows that the effect of novelty on the intention to use smart devices is also positive. So, Hypothesis 3, novelty is positively related to the intention to use smart healthcare devices, is also supported. However, the coefficient of convenience is 0.218 (*p* < 0.01). This means that price is not negatively related to the intention. Thus, Hypothesis 4, price is negatively related to the intention to use smart healthcare devices, is not supported. The coefficient of technological complexity is -0.157 (*p* < 0.05). Obviously, Hypothesis 5, technological complexity is negatively related to the intention to use smart healthcare devices, is supported by data. However, the coefficient of perceived privacy risk is -0.085 (ns). Therefore, Hypothesis 6, perceived privacy risk is negatively related to the intention to use smart healthcare devices, is not supported by samples. The results show that Hypothesis 4 and Hypothesis 6 are not supported. The possible reason is that the data collected from China are limited. Although we collected samples from several cities, the number of questionnaires is still not large. More questionnaires should be required to test the hypotheses in future.

RETRACTED

## 5. Theoretical and Public Policy Implications

Extending previous researches, this paper establishes a framework and identifies the factors affecting the acceptance of smart healthcare devices. Based on the samples from China, we test the effect of different factors on the intention to use smart devices. The results show there are several significant theoretical implications and public policy implications.

### 5.1. Theoretical Implications

This study contributes to the area of the smart healthcare industry as follows.

First, this study proposes a framework and identifies several factors that determine the intention to use smart healthcare devices. Previous studies mainly focus on the impact of various digital technologies on smart devices and the effect of smart healthcare devices on individuals' care and smart cities [8, 11, 12]. Few scholars study the acceptance of smart healthcare devices and the factors that influence the intention to use them. Considering that attributes of products, technological characteristics, and individual characteristics are studied independently, this study discuss them in a framework. This study identifies six factors, including the attributes of products or services (usefulness, convenience, novelty, and price of smart devices), technological complexity, and perceived privacy risk. By doing so, we address the theoretical gap of the acceptance of smart healthcare devices.

Second, this study examines the effects of different factors on the intention to use smart healthcare devices. Based on the samples from several cities in China, we find that usefulness, convenience, and novelty of smart devices are positively related to the intention to use these devices. In addition, technological complexity is negatively related to the intention. By doing so, this study explores different impacts of the attributes of products or services and technological complexity on the acceptance of smart healthcare devices. The findings further extend the understanding of the impacts of different factors on the intention to use the smart healthcare devices.

RETRACTED

### 5.2. Public Policy Implications

There are also several public policy implications.

First, governments should encourage the development of smart healthcare devices. Smart devices exploit different digital technologies such as machine learning and Internet of Things and provide intelligent services for users. This has greatly changed the traditional healthcare industry. Customers could utilize more convenient healthcare services at home. Everyone's health could be monitored at any time. This creates a smarter healthcare industry based on new technologies. However, smart healthcare devices are still in its infant stage. More resources and policies should be provided to develop this industry. For example, governments could reduce taxes and provide financial support for developing the new industry.

Second, governments should encourage the utilization of smart devices in multiple ways. Although it is important for individuals to use smart devices to monitor health conditions, the acceptance of smart devices is still not high. Government could publicize the usefulness of smart devices and let more people know the convenience of them. Especially for the smart healthcare devices that detect common diseases, their usefulness, convenience, and novelty should be widely reported. It is beneficial for users to recognize the smart devices.

Third, governments should reduce privacy risk through ways of established new institutions or laws. Perceived privacy risk is becoming an important obstacle for users. Unlike traditional healthcare, smart devices will collect users' information and data on health status [32]. Privacy information security is strongly concerned by users. How to avoid information disclosure and how to reduce privacy risk need to be addressed. This is a social problem and requires the intervention of governments. It is necessary to implement laws and regulations to prohibit the disclosure of personal privacy.

Finally, the health service system should strengthen the compatibility between smart healthcare devices and hospital services. There is a significant difference between the services provided by smart devices and the services provided by hospitals. The former emphasizes monitoring and prevention, which helps individuals manage physical health. It is beneficial to reduce the pressure of hospitals and increase the quality of hospital services. Obviously, it is valuable to improve the compatibility between smart healthcare devices and hospital services and strongly optimize the allocation of medical resources.

RETRACTED

## 6. Conclusions

The healthcare industry is strongly influenced by new digital technologies. In this context, this study creates a framework and explores determinants of the intention to use smart healthcare devices. Firstly, several factors that influence the intention to use smart devices were identified, including usefulness, convenience, novelty, price of smart devices, technological complexity, and perceived privacy risk. Secondly, a framework was established to examine the effect of these factors on the intention to use smart healthcare devices. The results show that there are different effects. The usefulness, convenience, novelty, and price have positive impacts on the intention to use smart devices. While the technological complexity variable shows negative influence on the intention. Third, theoretical implications and public policy implications were revealed on the basis of the findings. The results further extend previous researches in the area of healthcare industry.

## Figures and Tables

**Figure 1:** Research framework.

**Table 1:** Characteristics of samples.

Characteristics	*N*	Percentage
Age		
30 years or less	61	30.2
30–40 years	95	47.0
40–50 years	20	9.9
50–60 years	15	7.4
Above 60 years	11	5.4

Years of work		
3 years or less	55	27.2
3–5 years	19	9.4
5–10 years	49	24.3
Above 10 years	79	39.1

Family annual income		
30 000 RMB or less	23	11.4
30 000–60 000 RMB	27	13.4
60 000–100 000 RMB	37	18.3
100 000–150 000 RMB	41	20.3
Above 150 000 RMB	74	36.6

Educational background		
High school or below	21	10.4
Junior college	28	13.9
Bachelor's degree	76	37.6
Master or Ph.D. degree	77	38.1

**Table 2:** The results of descriptive statistics and Pearson correlation.

	1	2	3	4	5	6	7	8	9	10	11
Age	1										
Work experience	0.696^*∗∗∗*^	1									
Family income	−0.071	0.147^*∗*^	1								
Educational background	−0.306^*∗∗*^	−0.230^*∗∗*^	0.391^*∗∗∗*^	1							
Intention to use	−0.050	0.011	0.008	0.027	1						
Usefulness	−0.051	0.070	0.021	0.013	0.701^*∗∗∗*^	1					
Convenience	−0.019	0.087	0.004	−0.016	0.726^*∗∗∗*^	0.637^*∗∗∗*^	1				
Novelty	−0.098	−0.033	−0.067	0.017	0.553^*∗∗∗*^	0.620^*∗∗∗*^	0.632^*∗∗∗*^	1			
Price	0.074	0.103	−0.096	−0.081	0.299^*∗∗∗*^	0.224∗∗	0.301^*∗∗∗*^	0.405^*∗∗∗*^	1		
Technological complexity	0.003	−0.028	−0.172^*∗*^	−0.150^*∗*^	0.195^*∗∗*^	0.243^*∗∗∗*^	0.265^*∗∗∗*^	0.516^*∗∗∗*^	0.687^*∗∗∗*^	1	
Perceived privacy risk	−0.031	0.013	−0.032	−0.034	0.141^*∗*^	0.230^*∗*^	0.223^*∗∗*^	0.332^*∗∗∗*^	0.521^*∗∗∗*^	0.562^*∗∗∗*^	1
Mean	2.11	2.75	3.57	3.03	3.991	4.227	4.157	3.805	3.356	3.209	3.105
SD	1.087	1.233	1.392	0.969	1.073	0.950	0.924	1.018	1.060	1.041	1.171

Note： ^*∗*^*p* < 0.05； ^*∗∗*^*p* < 0.01； ^*∗∗∗*^*p* < 0.001.

RETRACTED

**Table 3:** The results of multiple linear regression analysis (MLR).

Variables	Model 1	Model 2
	Control variables
Age	−0.114	0.034
Work experience	0.100	−0.089
Family income	−0.025	0.015
Educational background	0.025	0.002

	Independent variables
Usefulness		0.371^*∗∗∗*^
Convenience		0.319^*∗∗∗*^
Novelty		0.143∗
Price		0.218^*∗∗*^
Technological complexity		−0.157^*∗*^
Perceived privacy risk		−0.085
*R* ^2^	0.007	0.592
Adj *R*^2^	−0.013	0.571
F value	0.363	27.731^*∗∗∗*^

Note：^*∗*^*p* < 0.05； ^*∗∗*^*p* < 0.01； ^*∗∗∗*^*p* < 0.001.

## Data Availability

The data used to support the findings of this study are available from the corresponding author upon request.

## References

[1] Nambisan S. (2017). Digital entrepreneurship: toward a digital technology perspective of entrepreneurship. *Entrepreneurship: Theory and Practice*.

[2] Bryndin E. (2018). Directions of development of industry 4.0, digital technology and social economy. *American Journal of Information Science and Technology*.

[3] Li W., Chai Y., Khan F. (2021). A comprehensive survey on machine learning-based big data analytics for IoT-enabled smart healthcare system. *Mobile Networks and Applications*.

[4] Shan B., Pu Y., Chen B., Lu S. (2021). New technologies’ commercialization: the roles of the leader’s emotion and incubation support. *Frontiers in Psychology*.

[5] Lee S. M., Lee D. H. (2021). Opportunities and challenges for contactless healthcare services in the post-COVID-19 era. *Technological Forecasting and Social Change*.

[6] Papa A., Mital M., Pisano P., Guiduice M. D. (2020). E-health and wellbeing monitoring using smart healthcare devices: an empirical investigation. *Technological Forecasting and Social Change*.

[7] Li Y., Shan B., Li B., Liu X., Pu Y. (2021). Literature review on the applications of machine learning and blockchain technology in smart healthcare industry: a bibliometric analysis. *Journal of Healthcare Engineering*.

[8] Baker S. B., Xiang W., Atkinson I. (2017). Internet of things for smart healthcare: technologies, challenges, and opportunities. *IEEE Access*.

[9] Tian S., Yang W., Grange J. M. L., Wang P., Huang W., Ye Z. (2019). Smart healthcare: making medical care more intelligent. *Global Health Journal*.

[10] Chui K., Alhalabi W., Pang S., Pablos P., Liu R., Zhao M. (2017). Disease diagnosis in smart healthcare: innovation, technologies and applications. *Sustainability*.

RETRACTED

[11] Sawyer J. (2020). Wearable internet of medical things sensor devices, artificial intelligence-driven smart healthcare services, and personalized clinical care in COVID-19 telemedicine. *American Journal of Medical Research*.

[12] Oueida S., Aloqaily M., Ionescu S. (2019). A smart healthcare reward model for resource allocation in smart city. *Multimedia Tools and Applications*.

[13] Tariq N., Qamar A., Asim M., Khan F. A. (2020). Blockchain and smart healthcare security: a survey. *Procedia Computer Science*.

[14] Magni D., Scuotto V., Pezzi A., Guiduice M. D. (2021). Employees’ acceptance of wearable devices: towards a predictive model. *Technological Forecasting and Social Change*.

[15] Sahut J.-M., Iandoli L., Teulon F. (2021). The age of digital entrepreneurship. *Small Business Economics*.

[16] Yang H., Yu J., Zo H., Choi M. (2016). User acceptance of wearable devices: an extended perspective of perceived value. *Telematics and Informatics*.

[17] Kim K. J., Shin D.-H. (2015). :An acceptance model for smart watches. *Internet Research*.

[18] Park E. (2020). User acceptance of smart wearable devices: an expectation-confirmation model approach. *Telematics and Informatics*.

[19] Ryu I., Choi H.-R. (2008). The effect of social influence on flow, perceived usefulness and intention to use in online community. *Journal of Information Systems*.

[20] Kim C., Mirusmonov M., Lee I. (2010). An empirical examination of factors influencing the intention to use mobile payment. *Computers in Human Behavior*.

[21] Kuo Y.-F., Yen S.-N. (2009). Towards an understanding of the behavioral intention to use 3G mobile value-added services. *Computers in Human Behavior*.

[22] Berry L. L., Seiders K., Grewal D. (2002). Understanding service convenience. *Journal of Marketing*.

[23] Hsu H., Chang Y. (2013). Extended TAM model: impacts of convenience on acceptance and use of Moodle. *Online Submission*.

[24] Amara N., Landry R., Becheikh N., Ouimet M. (2008). Learning and novelty of innovation in established manufacturing SMEs. *Technovation*.

[25] Koc T., Bozdag E. (2017). Measuring the degree of novelty of innovation based on Porter’s value chain approach. *European Journal of Operational Research*.

[26] Flor M. L., Cooper S. Y., Oltra M. J. (2018). External knowledge search, absorptive capacity and radical innovation in high-technology firms. *European Management Journal*.

[27] Sharma R., Yetton P. (2007). The contingent effects of training, technical complexity, and task interdependence on successful information systems implementation. *MIS Quarterly*.

RETRACTED

[28] Puddicombe M. S. (2012). Novelty and technical complexity: critical constructs in capital projects. *Journal of Construction Engineering and Management*.

[29] Antoniadis D. N., Edum-Fotwe F. T., Thorpe A. (2011). Socio-organo complexity and project performance. *International Journal of Project Management*.

[30] Ignatius J., Leen J. Y. A., Ramayah T., Hin C. K., Jantan M. (2012). The impact of technological learning on NPD outcomes: the moderating effect of project complexity. *Technovation*.

[31] Grande D., Marti X. L., Feuerstein-Simon R. (2020). Health policy and privacy challenges associated with digital technology. *JAMA Network Open*.

[32] Klobas J. E., McGill T., Wang X. (2019). How perceived security risk affects intention to use smart home devices: a reasoned action explanation. *Computers & Security*.

[33] Hiranandani V. (2011). Privacy and security in the digital age: contemporary challenges and future directions. *International Journal of Human Rights*.

[34] Alsabawy A. Y., Cater-Steel A., Soar J. (2016). Determinants of perceived usefulness of e-learning systems. *Computers in Human Behavior*.

[35] Nieto M. J., Santamaría L. (2007). The importance of diverse collaborative networks for the novelty of product innovation. *Technovation*.

